# Monocyte-to-Lymphocyte Ratio Was an Independent Factor of the Severity of Spinal Tuberculosis

**DOI:** 10.1155/2022/7340330

**Published:** 2022-05-20

**Authors:** Liyi Chen, Chong Liu, Tuo Liang, Zhen Ye, Shengsheng Huang, Jiarui Chen, Xuhua Sun, Ming Yi, Jie Jiang, Tianyou Chen, Hao Li, Wuhua Chen, Hao Guo, Yuanlin Yao, Shian Liao, Chaojie Yu, Shaofeng Wu, Binguang Fan, Zhaoping Gan, Xinli Zhan

**Affiliations:** ^1^Spine and Osteopathy Ward, Guangxi Medical University First Affiliated Hospital, Nanning, Guangxi Province, China; ^2^Department of Hematology, Guangxi Medical University First Affiliated Hospital, Nanning, Guangxi Province, China

## Abstract

**Purpose:**

The purpose was to explore the relationship between monocyte-to-lymphocyte ratio (MLR) and the severity of spinal tuberculosis.

**Methods:**

A total of 1,000 clinical cases were collected, including 496 cases of spinal tuberculosis and 504 cases of nonspinal tuberculosis. Laboratory blood results were collected, including C-reactive protein (CRP), erythrocyte sedimentation rate (ESR), white blood cells (WBC), hemoglobin (HGB), platelets (PLT), neutrophil count, percentage of neutrophils, lymphocyte count, percentage of lymphocytes, monocyte count, percentage of monocytes, MLR, platelets -to- monocyte ratio (PMR), platelets -to- lymphocyte ratio (PLR), neutrophil -to- lymphocyte ratio (NLR), and platelets -to- neutrophil ratio (PNR). The statistical parameters analyzed by the Least Absolute Shrinkage and Selection Operator (LASSO) and receiver-operating characteristic (ROC) curves were used to construct the nomogram. The nomogram was assessed by C-index, calibration curve, ROC curve, and decision curve analysis (DCA) curve.

**Results:**

The C-index of the nomogram in the training set and external validation set was 0.801 and 0.861, respectively. Similarly, AUC was 0.801 in the former and 0.861 in the latter. The net benefit of the former nomogram ranged from 0.1 to 0.95 and 0.02 to 0.99 in the latter nomogram. Furthermore, there was a correlation between MLR and the severity of spinal tuberculosis.

**Conclusion:**

MLR was an independent factor in the diagnosis of spinal tuberculosis and was associated with the severity of spinal tuberculosis. Additionally, MLR may be a predictor of active spinal tuberculosis.

## 1. Introduction

Tuberculosis poses a threat to human health all over the world and a huge economic burden on the people [1]. The incidence of spinal tuberculosis remains high, accounting for about 1%-3% of all tuberculosis [2]. Spinal tuberculosis is the most common type of extrapulmonary tuberculosis, accounting for 50% of skeletal tuberculosis [3]. Various examination methods have different limitations for the diagnosis of tuberculosis. The positive rates of acid-fast staining of sputum smears are usually used to diagnose tuberculosis. However, tuberculosis is easily missed due to the low sensitivity of the positive rate of acid-fast bacilli [4]. Although the culture of Mycobacterium tuberculosis is the gold standard for the diagnosis of tuberculosis, it cannot be used as an early diagnosis due to the low detection rate and long bacterial culture time [5]. In addition, the positive rate of spinal tuberculosis bacterial culture is only 44.39% reported in the literature [6]. Despite the rapid development of genetic testing, the positive rate of Mycobacterium tuberculosis DNA is only 66.67% [4]. Spinal tuberculosis is often diagnosed by pathological examination, but the sensitivity of histopathology of spinal tuberculosis ranges from 40.8% to 56.5% [7]. MLR has been reported in the literature as a predictor of tuberculosis diagnosis [8]. However, whether MLR can be used as a predictor in the diagnosis of spinal tuberculosis has not been reported.

MLR is closely associated with the expression of inflammatory factors in many diseases. Mehmet et al.'s study showed that MLR was not only positively correlated with microalbuminuria but also was determined as an independent factor of diabetic kidney injury by logistic regression analysis [9]. Aktas et al. found that MLR was involved in the inflammatory process of hepatic steatosis, and MLR was significantly higher in the hepatic steatosis group than in the control group [10]. MLR was significantly higher in irritable bowel syndrome, which may be a new inflammatory marker for irritable bowel syndrome diagnosed by laboratory examination [11]. In addition, MLR as an inflammatory marker was significantly different between colorectal cancer with and without metastasis, which may predict colorectal cancer metastasis [12]. Interestingly, COVID-19 is widespread around the world, and MLR as a marker of hematologic inflammation is a predictor involving diagnosis and clinical prognosis of the COVID-19 infection [13]. We hypothesized that MLR is also responsible for inflammatory factors in spinal tuberculosis.

ESR and CRP are usually highly expressed in inflammatory diseases and are used to assess the degree of infection of the disease [14]. Increasing ESR during treatment indicates severe spinal tuberculosis and poor prognosis [15]. CRP is as high as 41.9 mg/L before surgery for severe spinal tuberculosis and ESR is as high as 51.4 mm/h [16]. MLR has been confirmed as an inflammation marker in tuberculosis, and high levels of MLR are associated with severe tuberculosis [17]. However, the findings of Van et al. did not support the hypothesis that MLR was associated with tuberculin skin test positivity [18]. There are still contradictions in the association between MLR and tuberculosis. Furthermore, the association between MLR and the severity of spinal tuberculosis has not been reported.

In this paper, a total of 1,000 clinical data are collected, including training set data and external validation set data. We mainly discussed the diagnosis of MLR in spinal tuberculosis and the relationship between MLR and the severity of spinal tuberculosis. Furthermore, we also explored MLR as a predictor of active spinal tuberculosis.

## 2. Materials and Methods

### 2.1. Patients

All written consents were obtained from patients with spinal tuberculosis. The inclusion criteria for spinal tuberculosis cases were as follows: (1) diagnosed with spinal tuberculosis by postoperative pathological examination. (2) No disease that affected blood tests. (3) Complete information. The exclusion criteria for spinal tuberculosis cases were as follows: (1) denied spinal tuberculosis by postoperative pathological examination. (2) Had diseases that affected blood tests. (3) Existence of immune-related diseases. Active spinal tuberculosis was defined based on moderate to severe dysfunction. This article was approved by the Ethics Committee of the First Affiliated Hospital of Guangxi Medical University.

### 2.2. Data Collection

Clinical data were collected from our hospital's electronic medical record database from June 2012 to June 2021. 1000 clinical data were collected. These data were divided into a training set (700 cases) and an external validation set (300 cases) according to different periods. General information was collected, including gender, age, and body mass index (BMI). Laboratory blood results were collected, including CRP, ESR, WBC, HGB, PLT, neutrophil count, percentage of neutrophils, lymphocyte count, percentage of lymphocytes, monocyte count, percentage of monocytes, MLR, PMR, PLR, NLR, and PNR. The clinical score was evaluated by two senior specialist physicians, including ODI, VAS, and ASIA score.

### 2.3. Statistical Analysis

R software (version 4.1.1) and GraphPad Prism software (version 8.0) were used in this article. *T*-test was used to compare the two sets of data. The one-way ANOVA test was used to compare multiple sets of data. LASSO regression selected parameters with nonzero coefficients to obtain optimal lambda. Then, the parameters with AUC>0.6 were selected by the ROC curve. The predictive ability and accuracy of the nomogram were assessed by the C-index, calibration curve, ROC curve, and DCA curve. The external verification method further evaluated the predictive ability of the nomogram. Correlation analysis of data with normal distribution was used Pearson test, while Spearman test was used for data with non-normal distribution. All continuous variables were represented by mean ± standard deviation (SD). *P* less than 0.05 was defined as a statistical difference.

## 3. Results

### 3.1. The Diagnostic of MLR in Spinal Tuberculosis

700 clinical cases were collected to construct the training set, including 347 cases of spinal tuberculosis (Figures 1–3) and 353 cases of nonspinal tuberculosis (Figures 4–6). There were statistically different parameters between the two groups, including gender, age, BMI, ESR, WBC, HGB, PLT, neutrophil count, lymphocyte count, percentage of lymphocytes, percentage of monocytes, MLR, PLR, NLR, and PNR (Table 1). These parameters were included in the LASSO regression analysis (Figures 7(a) and 7(b)). The optimal lambda and nonzero coefficient parameters were selected by LASSO regression and were included in the ROC analysis (Figure 7(c)). In the training set, the parameters with AUC greater than 0.6 in the ROC curve were age (AUC =0.735), PLR (AUC =0.642), MLR (AUC =0.663), and percentage of monocytes (AUC =0.652). Similarly, the AUC of these parameters in the external validation set was 0.801, 0.706, 0.737, and 0.687, respectively (Figure 7(d)). These parameters were used to construct a nomogram. The predictive ability of the nomogram ranged from 0.01 to 0.99 in the training set (Figure 8). Similarly, the nomograms in the external validation set had the same predictive ability (Figure 9). The C-index in the training set was 0.801 and that was 0.861 in the external validation set. The observations in the calibration curve were highly similar to the ideal values, whether in the training set (Figure 10(a)) or the external validation set (Figure 10(b)). AUC was 0.801 in the training set (Figure 10(c)) and that was 0.861 in the external validation set (Figure 10(d)). The net benefit of this nomogram ranged from 0.1 to 0.95 in the training set (Figure 10(e)). Similarly, the benefit rate was also very high in the external verification set, ranging from 0.02 to 0.99 (Figure 10(f)).

### 3.2. MLR Was Closely Related to the Severity of Spinal Tuberculosis

496 cases of spinal tuberculosis were included. Cases were divided into high ODI group (score≥20) and low ODI group (score<20) according to the ODI score. There were statistically different parameters between the two groups, including age, ESR, HGB, percentage of neutrophils, lymphocyte count, percentage of lymphocytes, MLR, PLR, and NLR (Table 2). The MLR of the high ODI group was significantly higher than that of the low ODI group (Figure 11(a)). Cases were divided into low VAS group (score≤7) and high VAS group (score>7) according to the VAS score. There were statistically different parameters between the two groups, including age, PLR, and MLR. The MLR of the high VAS group was significantly higher than that of the low VAS group (Figure 11(b)). Cases were divided into five grades according to the ASIA classification. Parameters that were statistically different in ASIA included age, ESR, percentage of monocytes, and MLR (Figure 11(c)). MLR was related to ESR (Figure 11(d)) and CRP (Figure 11(e)). ESR was higher in the high ODI score group than in the low ODI score group (Figure 12(a)). Similarly, the level of ESR was statistically different in ASIA (Figure 12(c)). However, the level of ESR was not statistically different between the high VAS score group and the low VAS score group (Figure 12(b)). In the statistical analysis of ODI score, VAS score, and ASIA, there was no statistical difference in CRP level (Figure 12).

### 3.3. MLR as a Predictor of Active Spinal Tuberculosis

Active spinal tuberculosis was defined based on moderate to severe dysfunction. Parameters with statistical differences were included in the ROC curve analysis, including age, ESR, HGB, percentage of neutrophils, lymphocyte count, percentage of lymphocytes, MLR, PLR, and NLR. Parameters with AUC>0.6 were selected to construct the nomogram, including age, percentage of lymphocytes, MLR, and PLR (Figure 13(a)). The ability of the nomogram to predict active spinal tuberculosis ranged from 0.1 to 0.9 (Figure 13(b)). The observed value and the ideal value were consistent in the calibration curve (Figure 13(c)). AUC was 0.69 by ROC curve analysis (Figure 13(d)).

## 4. Discussion

The incidence of spinal tuberculosis in newborns has increased from 14% to 45.2%, posing a huge threat to humans [1, 19, 20]. Despite the rapid advancement of modern experimental technology, the positive detection rate of spinal tuberculosis is still not high. Diagnosis of spine tuberculosis usually uses the following methods: acid-fast tuberculosis smear, acid-fast tuberculosis DNA test, culture of mycobacterium tuberculosis, immunohistochemistry. However, the diagnostic value of MLR in spinal tuberculosis has not been reported.

MLR is significantly expressed in many diseases. MLR was used as a predictor of prostate cancer diagnosis and the AUC was 0.852 [21]. MLR>0.35 was associated with the overall survival rate of glioma patients [22]. High expression of MLR was detected in inflammatory diseases. High MLR expression was associated with mortality in acute respiratory distress syndrome [23]. MLR was significantly higher in patients with advanced knee synovitis than in early patients [23]. Our study found that MLR in the training set was statistically different between spinal tuberculosis and nonspinal tuberculosis. MLR was used as a predictor of spinal tuberculosis diagnosis, and its AUC was 0.663 by ROC curve analysis. The results of Sukson et al. showed that MLR was used as a predictor in the diagnosis of tuberculous pleuritis and the AUC was 0.91 [24]. Monocytes promoted the expression level of immune checkpoints and lead to latent tuberculosis infection [25]. MLR may affect the immune response of tuberculosis patients during the process of mycobacterium tuberculosis replication and progression to tuberculosis [26–28].

The severity of spinal tuberculosis had been reported to be associated with vitamin D receptor (VDR), osteopontin (OPN), and bone morphogenetic protein-4 (BMP-4) gene polymorphism [29]. Osteopontin mediated inflammation by regulating immune cells [30]. Our results found that MLR was associated with the severity of spinal tuberculosis. Osteopontin might have been involved in regulating MLR to promote the progression of spinal tuberculosis. A previous study also reported that the concentration of OPN in tuberculosis plasma was higher than that of healthy patients [31]. VDR was associated with the clinical severity of spinal tuberculosis [29]. It may be that VDR regulated the expression of multiple genes in monocytes [32]. MLR was closely related to the severity of the disease by promoting the activation of macrophages [33]. The results of our study were consistent with the finding that MLR was a marker of the severity of spinal tuberculosis.

ESR and CRP were used as inflammatory markers, usually used to assess the degree of inflammation of the disease [34]. In multidrug-resistant tuberculosis, ESR and CRP were as high as 62.03 mm/h and 83.24 mg/L, respectively, which were significantly higher than the ESR (37.20 mm/h) and CRP (50.02 mg/L) levels in drug-susceptible tuberculosis [35]. The expression of CRP was significantly increased in patients with advanced tuberculosis, but it lacked value in the diagnosis of early tuberculosis [36–38]. However, ESR and CRP also increased significantly in community-acquired pneumonia [39]. This made the diagnosis of spinal tuberculosis combined with community-acquired pneumonia more difficult. Our research showed that ESR and CRP had little contribution to the diagnosis of spinal tuberculosis and the severity of the disease. Our findings provided a distinction between the diagnosis of spinal tuberculosis and community-acquired pneumonia.

MLR had been reported as a marker for active diseases, such as systemic lupus erythematosus [40]. MRL had also been reported to increase expression levels in active gout [33]. Monocytes promoted the release of inflammatory mediators after pathogen invasion, and then transform into macrophages to participate in the immune response [41]. Inflammation was associated with low lymphocyte count [42]. Therefore, the increase in monocyte count and the decrease in lymphocyte count in inflammatory diseases lead to the imbalance of the MLR. Our findings also found that increased MLR was associated with the diagnosis of spinal tuberculosis, clinical severity, and active spinal tuberculosis.

In addition, PLR is also a marker of inflammation and is significantly expressed in a variety of diseases. Mehmet et al.'s study showed that PLR as an inflammatory factor was significantly higher in advanced fibrosis 119 (61-1547) % than in mild fibrosis 99.5 (36-259) %, with a significant difference between the two groups [43]. Hamdi et al.'s study showed that PLR was positively correlated with CRP and ESR in the thyroid conditions, which could predict the thyroid conditions with high uptake or normal uptake [44]. The expression of PLR in malignant thyroid nodules was higher than that in benign thyroid nodules, and there was a positive correlation with TSH [45]. In addition, PLR expression was significantly higher in diabetes mellitus than in healthy patients, and there was a positive correlation between PLR and HbA1c [46]. Similarly, we also found that PLR, as an inflammatory factor, was significantly higher in spinal tuberculosis than in nonspinal tuberculosis in this study (*P* < 0.001). However, the AUC of MLR (0.663) in diagnosing spinal tuberculosis was higher than that of PLR (0.642) in the training set. The former (0.737) is also higher than the latter (0.706) in the verification set.

However, this study still had some limitations. (1) This topic was single-center research. (2) Blood tests were only collected at a single time point, and blood tests at multiple time points were more convincing.

## 5. Conclusion

MLR as an independent factor was associated with the diagnosis of spinal tuberculosis and the severity of spinal tuberculosis. Furthermore, MLR may be a predictor of active spinal tuberculosis.

## Figures and Tables

**Figure 1:** X-ray examination of a patient with spinal tuberculosis. The arrow points to the location of the lesion. (a) X-ray image in posterior-anterior position. (b) X-ray image in lateral position.

**Figure 2:** CT examination of a patient with spinal tuberculosis. The arrow points to the location of the lesion. (a) CT image in sagittal position. (b) CT image in coronal position. (c) CT image in cross-section.

**Figure 3:** MRI examination of a patient with spinal tuberculosis. The arrow points to the location of the lesion. (a) MRI image in the sagittal T1 sequence. (b) MRI image in the sagittal T2 sequence. (c) MRI image of T2 lipid compression sequence in sagittal position. (d) MRI image in coronal position. (e) MRI image in cross-section.

**Figure 4:** X-ray examination of a patient with nonspinal tuberculosis. The arrow points to the location of the lesion. (a) X-ray image in posterior-anterior position. (b) X-ray image in lateral position.

**Figure 5:** CT examination of a patient with nonspinal tuberculosis. The arrow points to the location of the lesion. (a) CT image in sagittal position. (b) CT image in coronal position. (c) CT image in cross-section.

**Figure 6:** MRI examination of a patient with nonspinal tuberculosis. The arrow points to the location of the lesion. (a) MRI image in the sagittal T1 sequence. (b) MRI image in the sagittal T2 sequence. (c) MRI image of T2 lipid compression sequence in sagittal position. (d) MRI image in coronal position. (e) MRI image in cross-section.

**Figure 7:** LASSO regression analysis and ROC curve. (a) Nonzero coefficient parameters were selected by LASSO regression. (b) The parameters with optimal lambda were selected by LASSO regression. (c) The ROC curve of the training set. (d) The ROC curve of the external validation set.

**Figure 8:** The nomogram for the diagnosis of spinal tuberculosis in the training set.

**Figure 9:** The nomogram for the diagnosis of spinal tuberculosis in the external validation set.

**Figure 10:** Evaluate the model in the training set and external validation set. (a) Calibration curve in the training set. (b) Calibration curve in the external validation set. (c) ROC curve in the training set. (d) ROC curve in the external validation set. (e) DCA curve in the training set. (f) DCA curve in the external validation set.

**Figure 11:** The relationship between MLR and the severity of spinal tuberculosis. (a) ODI score. (b) VAS score. (c) ASIA. (d) Correlation between MLR and ESR. (e) Correlation between MLR and CRP.

**Figure 12:** (a–c) The relationship between ESR and the severity of spinal tuberculosis. (a) ODI score. (b) VAS score. (c) ASIA. (d–f) The relationship between CRP and the severity of spinal tuberculosis. (d) ODI score. (e) VAS score. (f) ASIA.

**Figure 13:** The nomogram and evaluation of active spinal tuberculosis. (a) ROC curve. (b) The nomogram for predicting active spinal tuberculosis. (c) The calibration curve of the predictive model. (d) The ROC curve of the predictive model.

**Table 1:** Comparison of clinical data in spinal tuberculosis and nonspinal tuberculosis.

Characteristics	Nonspinal tuberculosis (*N* =353)	Spinal tuberculosis (*N* =347)	*P*-value
Gender			
Female	46 (13%)	145 (42%)	<0.001
Male	307 (87%)	202 (58%)	
Age			
Mean ± SD	35.4 ± 10.4	49.4 ± 17.3	<0.001
BMI			
Mean ± SD	24.6 ± 9.00	20.5 ± 3.15	<0.001
ESR			
Mean ± SD	30.9 ± 22.3	39.3 ± 25.0	<0.001
CRP			
Mean ± SD	31.0 ± 40.5	31.1 ± 40.4	0.974
WBC			
Mean ± SD	8.23 ± 2.04	7.30 ± 2.76	<0.001
HGB			
Mean ± SD	132 ± 17.7	120 ± 17.7	<0.001
PLT			
Mean ± SD	318 ± 96.7	303 ± 104	0.039
Percentage of neutrophils			
Mean ± SD	0.630 ± 0.0972	0.628 ± 0.123	0.746
Neutrophil count			
Mean ± SD	5.27 ± 1.82	4.71 ± 2.42	<0.001
Percentage of lymphocytes			
Mean ± SD	0.262 ± 0.0836	0.237 ± 0.106	<0.001
Lymphocyte count			
Mean ± SD	2.09 ± 0.695	1.64 ± 0.843	<0.001
Monocyte count			
Mean ± SD	0.645 ± 0.248	0.652 ± 0.291	0.74
Percentage of monocytes			
Mean ± SD	0.0790 ± 0.0252	0.0960 ± 0.0579	<0.001
PMR			
Mean ± SD	541 ± 201	528 ± 242	0.458
MLR			
Mean ± SD	0.332 ± 0.153	0.487 ± 0.323	<0.001
PLR			
Mean ± SD	167 ± 74.6	228 ± 137	<0.001
NLR			
Mean ± SD	2.84 ± 1.68	3.69 ± 3.20	<0.001
PNR			
Mean ± SD	66.5 ± 30.2	75.3 ± 35.8	<0.001

**Table 2:** Comparison of clinical data in ODI score <20 and ODI score ≥20.

Characteristics	ODI<20 (*N* =329)	ODI ≥20 (*N* =167)	*P*-value
Gender			
Female	135 (41%)	64 (38%)	0.628
Male	194 (59%)	103 (62%)	
Age			
Mean ± SD	46.9 ± 17.4	56.7 ± 15.7	<0.001
BMI			
Mean ± SD	20.5 ± 3.34	20.4 ± 2.68	0.639
ESR			
Mean ± SD	38.5 ± 24.2	48.1 ± 39.6	0.004
CRP			
Mean ± SD	28.7 ± 38.2	32.9 ± 42.0	0.279
WBC			
Mean ± SD	7.26 ± 2.80	7.41 ± 2.88	0.561
HGB			
Mean ± SD	121 ± 16.7	117 ± 18.5	0.008
PLT			
Mean ± SD	299 ± 97.2	316 ± 112	0.082
Percentage of neutrophils			
Mean ± SD	0.624 ± 0.115	0.648 ± 0.134	0.045
Neutrophil count			
Mean ± SD	4.65 ± 2.47	4.98 ± 2.67	0.181
Percentage of lymphocytes			
Mean ± SD	0.245 ± 0.100	0.213 ± 0.111	0.002
Lymphocyte count			
Mean ± SD	1.69 ± 0.854	1.46 ± 0.752	0.002
Monocyte count			
Mean ± SD	0.634 ± 0.259	0.684 ± 0.317	0.078
Percentage of monocytes			
Mean ± SD	0.0934 ± 0.0444	0.105 ± 0.0822	0.081
PMR			
Mean ± SD	527 ± 226	527 ± 245	1
MLR			
Mean ± SD	0.456 ± 0.306	0.589 ± 0.427	<0.001
PLR			
Mean ± SD	215 ± 126	277 ± 196	<0.001
NLR			
Mean ± SD	3.51 ± 3.27	4.80 ± 7.89	0.044
PNR			
Mean ± SD	74.5 ± 31.9	76.9 ± 43.2	0.523

## Data Availability

The original contributions presented in the study are included in the article, further inquiries can be directed to the corresponding author/s.
